The article "CircAGFG1 Promotes Osteosarcoma Progression and Stemness by Competing with miR-302a-3p to Upregulate the Expression of LATS2" was retracted in 2023. Reasons: signs of a paper mill; compromised peer review; unreliable results or conclusions.

# CircAGFG1 Promotes Osteosarcoma Progression and Stemness by Competing with miR-302a-3p to Upregulate the Expression of LATS2

**DOI:** 10.1155/2022/6370766

**Published:** 2022-07-31

**Authors:** Tongchun Li, Guangjie Xing, Liangliang Lu, Xiangzhen Kong, Jinwei Guo

**Affiliations:** ^1^Department of Orthopedics, Changle County People's Hospital, Weifang 262400, Shandong, China; ^2^Department of Oncology, Shandong University of Traditional Chinese Medicine, Ji'nan 250355, Shandong, China; ^3^Department of Oncology, Sishui County People's Hospital, Jining 273299, Shandong, China; ^4^Department of Orthopedics, Chongqing University Jiangjin Hospital, Chongqing 402260, China

## Abstract

This study aimed to investigate the effect of circRNA (circAGFG1) on the proliferation, migration, invasion, and cell stemness of osteosarcoma cells by targeting miR-302a to regulate LATS2. The expression of circAGFG1 in osteosarcoma cells and normal osteoblasts was detected by real-time fluorescent quantitative PCR (RT-qPCR). Cell proliferation, clone formation, and invasion were detected by CCK-8, clone formation, and cell invasion assays. In vivo tumor formation assay was used to detect the effect of circAGFG1 on tumor growth. The expression level of circAGFG1 was upregulated in osteosarcoma cells. The downregulation of circAGFG1 inhibited the proliferation, invasion, and migration of osteosarcoma cells. The overexpression of circAGFG1 enhanced the stemness of osteosarcoma cells. CircAGFG1 was specifically bound to miR-302a to regulate the expression activity of miR-302a. MiR-302a specifically bound to the 3′UTR of LATS2 and inhibited the expression of LATS2. The overexpression of miR-302a reversed the effect of circAGFG1 on the proliferation, invasion, and migration of osteosarcoma cells. CircAGFG1 regulated the expression of LATS2 by miR-302a, thereby regulating the proliferation, migration, and invasion of osteosarcoma cells.

## 1. Introduction

Osteosarcomas arise from interosseous cells and are most common in long bones and in distal femur or proximal tibia [1]. Osteosarcoma is a primary malignant bone tumor. Osteosarcoma is characterized by a high degree of malignancy, small metastases before surgery, local recurrence, and a poor prognosis [2]. Patients treated with the combination of surgery and chemotherapy have 5-year survival rate of only 55%–65% [3]. With the development of gene therapy and other biological therapeutic techniques, new progress has been achieved in the comprehensive treatment of osteosarcoma [4–6].

CircRNAs (circRNAs) are a class of noncoding RNAs that are involved in the regulation of transcription and posttranscription gene expression [7]. CircRNA is closely related to the occurrence, progression, and treatment of tumors and also plays a significant role in the occurrence and progression of osteosarcoma [8–10]. Hence, circRNA may be a new breakthrough for the treatment of osteosarcoma. Liu et al. [11] found that circ-NT5C2 was upregulated in 52 pairs of osteosarcoma tissues and cell lines. Circ-NT5C2 silencing inhibited the proliferation and invasion of osteosarcoma cells and promoted the apoptosis of osteosarcoma cells. Circ-NT5C2 silencing inhibited tumor growth in vivo. Moreover, circRNA circAGFG1 promoted the progression of triple-negative breast cancer by regulating CCNE1 expression [12]. CircAGFG1 also promoted metastasis and xerosis in non-small-cell lung cancer [13] and colorectal cancer [14]. However, the role of circAGFG1 in osteosarcoma has not been reported yet.

CircRNA contains miRNA binding sites, allowing it to absorb miRNAs like a sponge, transform into competitive endogenous RNAs, isolate miRNAs, and inhibit their negative regulatory gene expression [15, 16]. Furthermore, the functional activity and expression level of target genes were improved. miRNA is expressed in human tissues and is related to normal physiological function and growth and development of the human body. miRNA regulates the growth, differentiation, metabolism, and other processes of tumor cells and is also a regulatory factor for the progression of various diseases [17]. The miR-302a gene is located on the miR-302 cluster on human chromosome 4 and is involved in the growth of embryonic stem cells and tumorigenesis [18]. MiR-302a is a downregulated miRNA found in colorectal cancer, ovarian cancer, and other tumors and inhibits the growth and metastasis of tumor cells [19]. However, the role of miR-302a in osteosarcoma and its relationship to the regulation of upstream and downstream target genes has not been reported. Large tumor suppressor factor (LATS2) is an important member of the LAST family [20]. The human chromosome is located in the 13q11-q12 region. LATS2 plays an important role in the regulation of cell cycle, check points, gene stability, inhibition of cell proliferation, and induction of apoptosis [21–23].

The underlying molecular mechanism of circRNAs in osteosarcoma remains unknown. In this study, we mainly discussed the expression of circAGFG1 in OS and conducted mechanistic studies to clarify its expression and clinical significance. Results provide an experimental basis for research of OS molecular markers and a new perspective for the clinical diagnosis and treatment of OS.

## 2. Methods

### 2.1. Cell Culture

NIH3T3, FOB, MG63, SaOS2, U2OS, and HOS cells were purchased from American Type Culture Collection (ATCC, Manassas, VA, USA) and treated with DMEM/F12 medium containing 10% FBS (Gibco, Life Technologies, Rockville, MD, USA) and supplemented with penicillin (100 U/mL) and streptomycin (100 U/mL) (Life Technologies, Rockville, MD, USA). U-2 OS was isolated and established from a moderately differentiated sarcoma of the tibia of a 15-year-old girl. The cells expressed insulin-like growth factor i, ii (IGF- i, IGF- ii) receptors, and osteosarcoma-derived growth factor (ODGF). HOS cells were isolated and established from osteosarcoma tissue of a 13-year-old white female. The cells were cultured in an incubator at a constant temperature of 37°C and 5% CO_2_. The medium was replaced with fresh complete medium every 3 days. When the cell density reached about 90%, the passage was performed at a ratio of 1 : 3.

### 2.2. Cell Transfection

Cells were spread on 12-well plates at a rate of 1 × 10^5^/well. When the cell density grew to about 70%, the plasmids of each group (50 nmol/L) were transfected into the cells according to the instructions of Lipofectamine 3000 transfection reagent (Life Technologies, Rockville, MD, USA). Lipofectamine 3000 was also used to transfect NC-mimics, miR-302a-3p mimics, NC (negative control)-siRNA, and LATS2 siRNA. After the transfected cells were placed in an incubator at 37°C and 5% CO_2_ for 48 h, cells in each group were collected for subsequent experiments.

### 2.3. Clone Formation

Cells with good growth were made into a cell suspension and seeded in cell culture plate at a rate of 1 × 10^3^/well. The plate was placed in an incubator at 37°C with 5% CO_2_ for about 14 days. The fluid was changed every 4 days, and cell growth was observed. The medium was removed, and the cells were washed with PBS three times. The cells were fixed with 4% paraformaldehyde for 20 min and stained with crystal violet (Solarbio, Beijing, China) for 5 min. Colonies with 30 or more cells were counted and photographed under a microscope.

### 2.4. Transwell Experiment

Matrigel stored at −20°C was melted overnight at 4°C and diluted with FBS-free medium on ice to a final concentration of 1 mg/mL. Each Transwell chamber was added with 100 *μ*L of diluted Matrigel (Thermo Fisher Scientific, Waltham, MA, USA) and placed in the incubator at 37°C for 5 h to dry into a gelatinous form. After cells were grown in each group, they were washed twice with PBS, subjected to trypsin digestion, and resuspended in medium without FBS to prepare cell suspension. The cell concentration was adjusted to 5 × 10^5^/mL. The cell suspension (100 *μ*L) was added to the upper compartment of the Transwell chamber, and complete medium was added to the lower compartment. The chamber was placed in the incubator at 37°C and 5% CO_2_ for 24 h. The compartment was removed, and the upper compartment medium was discarded. The samples were washed twice with PBS, fixed with 4% paraformaldehyde for 20 min, and stained with 0.1% crystal violet for 20 min. The upper unmigrated cells were carefully erased with a cotton swab and washed with PBS twice. Five fields of vision were selected under the microscope for cell observation and counting.

### 2.5. Determination of Cell Viability by CCK-8 Method

Cells were spread in 96-well plates at a density of 1 × 10^5^/mL. The culture was placed in the incubator at 37°C and 5% CO_2_. When the cell density grew to about 75%, the plasmids were transfected into each group. Five wells were set in each group, and the supernatant was removed after 48 h of culture. Each well received 100 *μ*L of a mixed culture medium (CCK-8 working medium to medium ratio of 1 : 10) (Beyotime, Shanghai, China) and was cultured in the incubator for 2 h. The absorbance (*A*) values of the cells in each well at 450 nm were read with a microplate analyzer.

### 2.6. QRT-PCR

Total RNA was extracted by TRIzol method. Reverse transcription was performed using One-Step Prime Script miRNA cDNA Synthesis (Takara Biotechnology Co., Ltd., Dalian, China). The reverse transcription system consisted of 1.0 *μ*g of total RNA, 2.0 *μ*L of 0.1% BSA, 10.0 *μ*L of 2 × miRNA Reaction Buffer Mix, 2.0 *μ*L of Prime Script RT Enzyme Mix, and RNase-free H_2_O to a total volume of 20 *μ*L. The reverse transcription procedure was as follows: 37°C, 60 min; 85°C, 5 min; and termination at 4°C. Real-time quantitative PCR was performed with SYBR Premix Ex Taq. The PCR procedure was as follows: 95°C, 10 s; 95°C, 5 s; 60°C, 20 s, 40 cycles. The following primers were used: circAGFG1, Forward: 5′-CCAGTTGTAGGTCGTTCTCAAG-3′, Reverse: 5′-TCACCCTGTGTGGTGGAT-3′; LATS2, Forward: 5′-TAGAGCAGAGGGCGCGGAAG-3′, Reverse: 5′-CCAACACTCCACCAGTCACAGA-3′; miR-302a, Forward: 5′-TAAGTGCTTCCATHTTGGTGA-3′, Reverse: 5′-TAAACCAAGTAAAATGGTCGA-3′. The upstream primer sequence of U6 is 5′-TTATGGGTCCTAGCCTGAC-3′, and the downstream primer sequence is 5′-CACTATTGCGGGCTGC-3′. The upstream primer of GAPDH is 5′-CAATGACCCCTTCATTGACC-3′, and the downstream primer is 5′-TTGATTTTGGAGGGATCTCG-3′. U6 and GAPDH were used as internal parameters. The relative expression of the target gene was calculated by 2^−△△CT^ method.

### 2.7. Xenograft Tumor Model

Six-week-old female BALB/c nude mice were purchased from Beijing Charles River Experimental Animal Technology Co., Ltd. Animal experiments were approved by the Animal Experiment Ethics Committee of Chongqing Jiangjin District Central Hospital and conducted in strict accordance with the operating norms. Stable cell lines were resuscitated and expanded to a concentration of 1 × 10^7^ cells/mL. Ultraclean table was disinfected with UV in advance, and the skin of nude mice was gently wiped with a cotton swab dipped in iodophor. The cells were gently mixed with a 1 mL syringe. The left side and axilla of nude mice were subcutaneously injected with 0.1 mL of stable cells. After the tumor cells were inoculated, the status of nude mice was observed every 2 days. Tumors began to appear in the axilla of nude mice about 5 days after the inoculation. Tumor size was measured every 3 days thereafter. After 21 days of tumor implantation, nude mice were euthanized with carbon dioxide in the euthanasia box. The chamber for euthanasia was filled with CO_2_ at a rate of 20% replacement volume per minute. When the animal does not move or breathe and its pupil dilates, shut off the CO_2_. Observation for another 3 min was conducted to ensure that the animal was dead. The tumor tissue was removed, labeled separately, weighed, and photographed. The lung tissue of the nude mice was placed in an EP tube along with 1 mL of precooled tissue fixation solution. The fixed tissue was used for HE staining. Other tumor tissues were used to extract RNA for testing.

### 2.8. HE Staining

The tissue fixed with paraformaldehyde was embedded in paraffin. Sequential sections were stained with hematoxylin–eosin (HE). The tissue was dewaxed with xylene I and II for 10 min, followed by 100% (I, II), 90%, 80%, and 70% alcohol for 5 mins each, and tap water for 5 min for three times. Hematoxylin was dyed for 5 min, and 5% acetic acid was differentiated for 1 min and rinsed with running water. Eosin was dyed for 1 min. Dehydration was conducted with 70%, 80%, 90%, and 100% alcohol 10 seconds each followed by xylene for 1 min. Neutral gum was dropped, and the tissue was observed and photographed under a microscope. Direct counting method was used to observe the number of lung metastases in nude mice.

### 2.9. Fluorescence In Situ Hybridization

A 10 mm × 10 mm glass slide was placed in a 24-well culture plate. Cells in the logarithmic growth phase were seeded into 24-well plates with a density of 6 × 10^3^ cells per well. The supernatant was removed after 24 h of culture, and the solution was fixed with paraformaldehyde at 4°C and 0.1% TritonX-100 was added. Prehybridization was performed at 37°C by adding prehybridization solution. The solution was added with a probe and hybridized at 42°C for 16–20 h. The sample was rinsed twice with sodium citrate buffer. DAPI fluorescent dye was dropped and stained in the section hybridization region for 10 min. After washing with phosphate buffer saline (PBS), the samples were observed under a fluorescence microscope.

### 2.10. Double-Luciferase Reporter Gene Detection

The Starbase website predicts the potential target genes of circAGFG1. TargetScan database was used to analyze the potential target genes of miR-302a. The circAGFG1 3′UTR fragment and LATS2 3′UTR fragment were amplified by PCR and cloned into the psiCHECK2 plasmid to construct ps-iCHECK2-circAGFG1-wt and LATS2-wt vectors. The point mutation kit was used to construct psiCHECK2-circAGFG1-mut and LATS2-mut vectors. The recombinant plasmid was transfected into the cells for 48 h. A dual-luciferase activity detection kit was used to determine the luciferase activity of the cells.

### 2.11. Statistical Analysis

SPSS 19.0 software (SPSS Inc., Chicago, IL, USA) was used to analyze data, and the results of at least three independent experiments were taken. Measurement data conforming to normal distribution are expressed as mean ± standard deviation. One-way analysis of variance followed by Tukey's multiple comparison test was used for comparison among multiple groups. Student's test was used for pairwise comparison between groups. *P* < 0.05 was considered statistically significant.

## 3. Results

### 3.1. circAGFG1 Promotes the Proliferation, Migration, Invasion, and Metastasis of Osteosarcoma Cells

To determine the role of circAGFG1 in osteosarcoma, we first detected its expression in osteosarcoma cells. The expression of circAGFG1 in osteosarcoma cell lines MG63, U2OS, SAOS2, HOS, and 143B was significantly higher than that in FOB and NIH3T3 cells (Figure 1(a)). The expression of circAGFG1 in U2OS and HOS cells was downregulated by shRNA transfection. Transfection efficiency was measured by real-time quantitative PCR at 48 h after transfection. The use of shRNA significantly reduced the circAGFG1 level in U2OS and HOS cells compared with empty vector cells (Figure 1(b)). U2OS and HOS cells were transfected after 48 h, and clone formation experiment was performed. The number of clones of U2OS and HOS cells in the experimental group was significantly lower than that in the control group, and the difference was statistically significant (Figure 1(c)). Hence, the downregulation of circAGFG1 expression can reduce the clonogenic ability of U2OS and HOS cells. The Transwell invasion test results showed that the number of transmembrane U2OS and HOS cells in the experimental group was significantly lower than that in the control group, and the difference was statistically significant (Figure 1(d)). As such, the downregulation of circAGFG1 expression can reduce the invasion ability of U2OS and HOS cells. CCK-8 experiments showed that the proliferation ability of U2OS and HOS cells was significantly reduced after circAGFG1 knockdown (Figure 1(e)).

## 4. Knocking down circAGFG1 Inhibited the Proliferation and Metastasis of Osteosarcoma Tumors

CircAGFG1 was stably knocked down in HOS cells, and tumor-bearing animal experiment was carried out in nude mice. After circAGFG1 knockdown, the tumor volume of HOS cells decreased compared with that in the control group, and the difference was statistically significant (Figure 2(a)). After sh-circAGFG1, the tumor weight of xenotransplantation was also smaller than that in the control group (Figure 2(b)). The tumor proliferation curve of the sh-circAGFG1 xenograft was smaller than that of the control group (Figure 2(c)). The expression of circAGFG1 in tumor tissues was detected by qRT-PCR. The use of lentiviral shRNA significantly reduced the circAGFG1 level compared with the cells with empty vectors (Figure 2(d)). The tumor metastasis rate of the sh-circAGFG1 xenograft was less than that of the control group (Figure 2(e)). Hence, the downregulation of circAGFG1 expression can reduce the proliferation and metastasis of osteosarcoma HOS cells.

### 4.1. Overexpression of circAGFG1 Enhanced the Stemness of Osteosarcoma Cells

The expression of circAGFG1 in U2OS and HOS cells was upregulated by transfection. Transfection efficiency was measured by real-time quantitative PCR at 48 h after transfection. The expression of circAGFG1 in U2OS and HOS cells transfected with overexpressed plasmid significantly increased compared with that in the control group, and the difference was statistically significant (Figure 3(a)). We also detected the changes in stem cell markers in U2OS and HOS cells by qRT-PCR after circAGFG1 overexpression. Experimental results showed that stemness markers CD133, SOX2, and CD90 on circAGFG1 were overexpressed in U2OS and HOS cells (Figures 3(b)–3(d)).

### 4.2. Regulatory Relationship among circAGFG1, miR-302a, and LATS2

The FISH assay showed that circAGFG1 was mainly located in the cytoplasm of osteosarcoma cells (Figure 4(a)). Starbase predicted binding sites between circAGFG1 and miR-302a (Figure 4(b)). The regulatory relationship between circAGFG1 and miR-302a was determined by dual-luciferase reporting system. The luciferase activity was significantly decreased in the psiCHECK2-circAGFG1-wt + miR-302a mimics group compared with that in the psiCHECK2-circAGFG1-wt + miR-302a NC-mimics group. Compared with the psiCHECK2-circAGFG1-mut + miR-302a NC-mimics group, luciferase activity had no significant change in the psiCHECK2-circAGFG1-mut + miR-302a mimics group (Figure 4(c)). The TargetScan website predicted that miR-302a and LATS2 had binding sites (Figure 4(d)). The dual-luciferase reporter gene assay results showed that compared with the pGL3-LATS2-wt + miR-302a NC-mimics group, the luciferase activity significantly decreased in the pGL3-LATS2-wt + miR-302a mimics group. No significant change in luciferase activity was detected in the PGL3-LATS2-Mut + miR-302a mimics group and PGL3-LATS2-Mut + miR-302a NC-mimics groups (Figure 4(e)). We further detected the expression of miR-302a-3p in tumor tissues by qRT-PCR. Compared with cells with empty vectors, the use of lentivirus shRNA significantly increased the level of miR-302a-3p (Figure 4(f)).

### 4.3. Correlation of circAGFG1, LATS2, and miR-302a-3p in Osteosarcoma

The RT-PCR results showed that the relative expression level of miR-302a increased in the miR-302a mimics group compared with that in the miR-302a NC-mimics group (Figure 5(a)). In addition, LATS2 siRNA decreased the expression of LATS2 in U2OS and HOS cells (Figure 5(b)). The proliferation rates of U2OS and HOS cells were significantly reduced upon stimulation by LATS2-siRNA or miR-302a-3p. However, circAGFG1 overexpression partially reduced the role of LATS2-siRNA or miR-302a-3p in U2OS and HOS cells (Figures 5(c) and 5(d)). The clone formation ability of U2OS and HOS cells was significantly reduced after stimulation by LATS2-siRNA or miR-302a-3p. However, circAGFG1 overexpression partially reduced the role of LATS2-siRNA or miR-302a-3p in U2OS and HOS cells (Figures 5(e) and 5(f)).

### 4.4. Expression of circAGFG1, LATS2, and miR-302a-3p in Osteosarcoma Cells and Their Relationship

The RT-PCR results showed that when circAGFG1 was knocked down in U2OS and HOS cells, the expression of LATS2 mRNA decreased compared with that in the control group (Figure 6(a)). After circAGFG1 was knocked down, the expression of miR-302a increased (Figure 6(b)). Compared with that in control cells, the expression level of miR-302a-3p was lower in stably transfected circAGFG1-overexpressed U2OS and HOS cells (Figure 6(c)). LATS2 was highly expressed in stably transfected circAGFG1-overexpressing U2OS and HOS cells compared with that in control cells (Figure 6(d)). The relative expression level of LATS2 mRNA decreased in the miR-302a mimics group compared with that in the miR-302a NC-mimics group (Figure 6(e)).

## 5. Discussion

Osteosarcoma is the most common primary malignant osteogenic bone tumor [24]. With the advent of the combination of preoperative neoadjuvant chemotherapy, surgery, and postoperative chemotherapy, the 5-year survival rate for patients with osteosarcoma has significantly increased [25]. However, the treatment of osteosarcoma has reached a bottleneck in recent decades [26]. Patients with metastasis have poor prognosis [27]. How to inhibit the metastasis of osteosarcoma is an urgent problem to be solved [28, 29].

The dysregulation of circRNA plays an important role in the occurrence and progression of osteosarcoma [30]. The abnormal expression of circRNA in osteosarcoma can cause the occurrence and progression of osteosarcoma [31–33]. For example, hsa_circ_0009910 acts as a sponge for miR-449a and upregulates functional target genes, leading to osteosarcoma [34]. Increasing number of studies have been conducted on the correlation between circRNA and tumor prognosis. Tumor prognostic indicators, such as tumor size, stage, and lymph node metastasis, showed varying degrees of correlation with some circRNAs. These circRNAs are differentially expressed in tumors, suggesting their prognostic significance. Li and Li [35] found that the upregulation of circ-0007534 was closely related to larger tumor diameter and lower differentiation degree in patients with osteosarcoma. In addition, patients with osteosarcoma and high circ-0007534 expression had shorter overall survival. Hence, circ-0007534 may play a key role in the regulation of the occurrence and progression of osteosarcoma and is an effective marker for predicting the prognosis of patients with osteosarcoma.

In this study, circAGFG1 was highly expressed in osteosarcoma cells. circAGFG1 affects the proliferation, invasion, and migration of osteosarcoma cells. To further verify whether the abnormal high expression of circAGFG1 is closely related to the invasion and migration of osteosarcoma cells, we selected siRNA to downregulate the expression of circAGFG1. We then used clone formation assay and Transwell assay to observe the changes in the stemness and migration ability of osteosarcoma cells. The downregulation of circAGFG1 expression could inhibit the stemness, invasion, and migration of osteosarcoma cells. Hence, circAGFG1 plays an oncogene role in the regulation of invasion and migration in osteosarcoma. Starbase was used to predict whether miR-302a is the target of circAGFG1. Studies have reported that miRNA is closely related to the occurrence and development of tumors. For example, miR-302a can inhibit the proliferation and invasion of thyroid cancer cells. CircRNAs have miRNA binding sites and can play a role as molecular sponges of miRNAs during tumor development. In this study, circAGFG1 regulated the expression of miR-302a, thereby affecting the proliferation, invasion, and migration of osteosarcoma cells. The TargetScan analysis and dual-luciferase reporter gene detection revealed that miR-302a could specifically bind to LATS2.

Studies on the regulatory mechanism of miRNAs found that miRNAs play various biological roles by targeting the expression of downstream target genes. In recent years, the expression and function of miR-302a in tumor tissues have attracted extensive attention. MiR-302a can inhibit the expression of drug-resistant proteins to improve the sensitivity of drug-resistant breast cancer cells to Adriamycin and can be used as a new target for the treatment of drug-resistant breast cancer [36]. The upregulation of miR-302a can inhibit the proliferation and invasion of colorectal cancer cells by regulating the MAPK and PI3K pathways and is an important target for the treatment of colorectal cancer [37]. Our experiment showed that the proliferation, invasion, and migration of osteosarcoma cells decreased after the upregulation of miR-302a expression. Hence, miR-302a plays an inhibitory role in the malignant phenotype of osteosarcoma cells and can inhibit the metastatic potential of osteosarcoma cells.

The Hippo signaling pathway is closely related to a variety of human malignant tumors, and LATS2, an important component of the signaling pathway, plays an important role in it. The LATS2 gene regulates cell cycle transformation by participating in a variety of cell signal transduction mechanisms, including pathways, signals, and genes. LATS2 can affect the proliferation and differentiation of tumor cells by regulating the balance of cell growth in the body. LATS2 is an important regulatory factor that promotes cancer progression and participates in tumorigenesis [38]. The overexpression of CCAT2 promoted the malignant progression of gastric cancer cells by upregulating LATS2 [39]. In the present study, circAGFG1 promoted the proliferation and cell stemness of osteosarcoma cells by inhibiting miR-302a-3p and upregulating the expression of LATS2.

The cancer-promoting mechanism of circAGFG1 needs to be further explored. In addition to regulating Mir-302A-3p/LATS2 axis, whether circAGFG1 has other target genes remains to be investigated. The downstream regulation mechanism of LATS2 was not determined in this study. Further research is needed for the clinical applications of the findings.

## 6. Conclusion

CircAGFG1 regulates the expression of LATS2 through miR-302a, thereby regulating the proliferation, invasion, and migration of osteosarcoma cells. This study suggests that circAGFG1 may be a potential therapeutic target for OS. However, the mechanism of action may be only one aspect, and the relationship among circAGFG1, miR-302a, and LATS2 needs to be further explored. This study provides a theoretical foundation for the application of circAGFG1 in clinical targeted therapy of osteosarcoma.

## Figures and Tables

**Figure 1:** circAGFG1 drives osteosarcoma cell proliferation, migration, invasion, and metastasis. (a) The expression of circAGFG1 in osteosarcoma cell lines was significantly higher than that of FOB and NIH3T3 cells. (b) Detection of transfection efficiency by qRT-PCR. Compared with cells with empty vectors, the use of lentiviral shRNA can significantly reduce the level of circAGFG1. (c) Clone formation assays in U2OS and HOS cells showed that the number of clones was reduced in circAGFG1 knockdown cells compared to control cells. (d) The Matrigel-coated Transwell experiment showed that, when circAGFG1 was knocked down, the invasion potential of U2OS and HOS was significantly reduced. (e) CCK-8 experiment showed that, after knocking down circAGFG1, the proliferation ability of U2OS and HOS was significantly reduced. ^*∗*^*P* < 0.05, ^*∗∗*^*P* < 0.01. NC: negative control. n.s.: not significant.

**Figure 2:** Knockdown of circAGFG1 inhibits tumor proliferation and metastasis of osteosarcoma. (a) Representative pictures of tumors of HOS cells with different expression levels of circAGFG1 in nude mice. (b) The weight of sh-circAGFG1 xenograft tumor is smaller than that of the control group. (c) The tumor proliferation curve of sh-circAGFG1 xenograft tumor is smaller than that of the control group. (d) Detection of circAGFG1 expression in tumor tissues by qRT-PCR. Compared with cells with empty vectors, the use of lentiviral shRNA can significantly reduce the level of circAGFG1. (e) The tumor metastases of sh-circAGFG1 xenograft tumors were smaller than those of the control group. ^*∗∗*^*P* < 0.01.

**Figure 3:** Overexpression of circAGFG1 enhances the stemness characteristics of osteosarcoma cells. (a) Detection of transfection efficiency by qRT-PCR. circAGFG1 is highly expressed in the transfected U2OS and HOS cells. (b) In U2OS and HOS cells, overexpression of circAGFG1 upregulated the expression of stemness marker CD133. (c) In U2OS and HOS cells, overexpression of circAGFG1 upregulated the expression of stemness marker SOX2. (d) In U2OS and HOS cells, overexpression of circAGFG1 upregulated the expression of stemness marker CD90. ^*∗∗*^*P* < 0.01.

**Figure 4:** circAGFG1 as a posttranscriptional regulator. (a) RNA FISH shows that circAGFG1 is mainly located in the cytoplasm of osteosarcoma cells. (b) The predicted potential binding site between circAGFG1 and miR-302a-3p. (c) The dual-luciferase reporter gene verifies the binding of circAGFG1 and miR-302a-3p. Luciferase activity in 293T cells when circAGFG1 WT or Mut vector is cotransfected with miR-302a-3p mimic or negative control. The miR-302a-3p mimic reduced the luciferase activity of the circAGFG1-WT reporter vector but did not reduce the luciferase activity of the empty vector or the mutant reporter vector. (d) The predicted potential binding site between miR-302a-3p and LATS2. (e) The dual-luciferase reporter gene verifies the binding of LATS2 to miR-302a-3p. Luciferase activity in 293T cells when LATS2 WT or Mut vector is cotransfected with miR-302a-3p mimic. The miR-302a-3p mimic reduced the luciferase activity of the LATS2 WT reporter gene vector but did not reduce the luciferase activity of the LATS2 mutant reporter gene vector. (f) Detection of miR-302a-3p expression in tumor tissues by qRT-PCR. Compared with cells with empty vectors, the use of lentivirus shRNA can significantly increase the level of miR-302a-3p. ^*∗∗*^*P* < 0.01. n.s.: not significant.

**Figure 5:** The correlation of circAGFG1, LATS2, and miR-302a-3p in osteosarcoma cell lines and xenograft tumors. (a) Detection of miR-302a-3p transfection efficiency in U2OS and HOS cells. (b) Detection of LATS2 transfection efficiency in U2OS and HOS cells. (c) U2OS cell proliferation test showed that the cell proliferation ability was significantly reduced in the cells mock-transfected with LATS2-siRNA or miR-302a-3p. The overexpression of circAGFG1 partially reduced the effect of LATS2-siRNA or miR-302a-3p in U2OS cells. (d) The results of cell proliferation assay in HOS cells are similar. (e) U2OS cell clone formation test showed that, in the cells mock-transfected with LATS2-siRNA or miR-302a-3p, the cell clone formation ability was significantly reduced. The overexpression of circAGFG1 partially reduced the effect of LATS2-siRNA or miR-302a-3p in U2OS cells. (f) The results of cell cloning assay in HOS cells are similar. (g) U2OS cell Transwell test showed that in the cells mock-transfected with LATS2-siRNA or miR-302a-3p, the cell migration ability was significantly reduced. The overexpression of circAGFG1 partially reduced the effect of LATS2-siRNA or miR-302a-3p in U2OS cells. (h) The results of cell Transwell assay in HOS cells are similar. ^*∗∗*^*P* < 0.01.

**Figure 6:** The expression of circAGFG1, LATS2, and miR-302a-3p in osteosarcoma cells and their relationship. (a) The LATS2 mRNA in cells knocked down circAGFG1 was significantly lower than that in control xenograft tumors. (b) The miR-302a-3p in circAGFG1 knockdown cells was significantly higher than that in the control. (c) Compared with control cells, LATS2 is highly expressed in the stably transfected circAGFG1 overexpressing U2OS and HOS cells. (d) Compared with control cells, miR-302a-3p is underexpressed in stably transfected circAGFG1 overexpressing U2OS and HOS cells. (e) In U2OS and HOS cells, overexpression of miR-302a-3p inhibits the expression of LATS2. ^*∗∗*^*P* < 0.01.

## Data Availability

The data used to support the findings of this study are available from the corresponding author upon request.
